# A complex evolutionary relationship between HHV-6A and HHV-6B

This article has been retracted.

**DOI:** 10.1093/ve/vez043

**Published:** 2019-10-20

**Authors:** Diego Forni, Rachele Cagliani, Mario Clerici, Uberto Pozzoli, Manuela Sironi

**Affiliations:** 1 Bioinformatics, Scientific Institute IRCCS E. Medea, Bosisio Parini, Lecco, Italy; 2 Department of Physiopathology and Transplantation, University of Milan, Milan, Italy; 3 IRCCS Fondazione Don Carlo Gnocchi, Milan, Italy

**Keywords:** HHV-6, Human betaherpesvirus, population structure, viral evolution, recombination

## Abstract

Human betaherpesviruses 6A and 6B (HHV-6A and HHV-6B) are highly prevalent in human populations. The genomes of these viruses can be stably integrated at the telomeres of human chromosomes and be vertically transmitted (inherited chromosomally integrated HHV-6, iciHHV6). We reconstructed the population structure of HHV-6 and we show that HHV-6A genomes diverged less than HHV-6B genomes from the ancestral common HHV-6A/B population. Analysis of ancestry proportions indicated that HHV-6A exogenous viruses and iciHHV-6A derived most of their genomes from distinct ancestral sources. Conversely, exogenous viral and iciHHV-6B populations were similar in terms of ancestry components, with no evident geographic structuring. Most HHV-6B genomes sampled to date derive from viral populations that experienced considerable drift. However, a population of HHV-6 exogenous viruses, currently classified as HHV-6B and sampled in New York state, formed a separate cluster (NY cluster) and harbored a considerable portion of HHV-6A-like ancestry. Recombination detection methods identified these viruses as interspecies recombinants, but phylogenetic reconstruction indicated that the recombination signals are due to shared ancestry. In analogy to iciHHV-6A, NY cluster viruses have high nucleotide diversity and constant population size. We propose that HHV-6A sequences and the NY cluster population diverged from an ancestral HHV-6A-like population. A relatively recent bottleneck of the NY (or a related) population with subsequent expansion originated most HHV-6B genomes currently sampled. Our findings indicate that the distinction between HHV-6A and -6B is not as clear-cut as previously thought. More generally, epidemiological and clinical surveys would benefit from taking HHV-6 genetic diversity into account.

## 1. Introduction

Human betaherpesviruses 6A and 6B (HHV-6A and HHV-6B) are members of the *Roseolovirus* genus, in the *Betaherpesviridae* subfamily. Initially described as viral variants, HHV-6A and -B are now formally recognized as distinct species by the ICTV (International Committee on Taxonomy of Viruses) and reportedly display about 90% interspecies genome sequence identity (Ablashi et al. 2014). HHV-6 genomes comprise a long unique region (∼145 kb) flanked by identical direct repeats (DR) (Krug and Pellett 2014). A variable number of perfect telomere-like repeat arrays are located at the right and left ends of the DRs and are thought to mediate viral integration into the host genome (Krug and Pellett 2014). In fact, unlike all other human herpesviruses, HHV-6A and HHV-6B can integrate and persist in the telomeric regions of host chromosomes (Luppi et al. 1993; Nacheva et al. 2008).

Primary infection with HHV-6B is extremely common and generally occurs before 24 months of age. The most common symptom is high fever and, although the course is usually benign, a minority of patients develops encephalitis (Hill and Zerr 2014; Tesini, Epstein, and Caserta 2014). For unknown reasons, the frequency of neurological complications varies with geography, being much higher in Japan than in the USA (Tesini, Epstein, and Caserta 2014). The epidemiology of HHV-6A is poorly described. When compared with HHV-6B, primary infection tends to occur later in life in Europe, America, and Asia; in sub-Saharan Africa, contrasting data on the prevalence of HHV-6A infection in infants were reported (Kasolo, Mpabalwani, and Gompels 1997; Bates et al. 2009; Tembo et al. 2015).

After primary infection, HHV-6 achieves latency, possibly by chromosomal integration in a small number of host cells (Arbuckle et al. 2010). Reactivation of latent HHV-6B represents a leading cause of central nervous system disease in transplant recipients (Hill and Zerr 2014).

HHV-6 chromosomal integration can also occur in the germ-line: in this case the viral genome is vertically transmitted from parent to child, behaving as a Mendelian trait (inherited chromosomally integrated HHV-6, iciHHV6) (Daibata et al. 1999; Tanaka-Taya et al. 2004; Kaufer and Flamand 2014). The proportion of iciHHV-6 carriers in the general population is 0.2–1%, with possible geographic differences both in overall frequency and in the relative proportion of HHV-6A and -6B integrations (Clark 2016; Tweedy et al. 2016).

Besides complicating the diagnosis of active HHV-6A/B infection, reactivation of iciHHV-6 was documented during pregnancy (Gravel, Hall, and Flamand 2013) and in an immunocompromised child (Endo et al. 2014). iciHHV-6 carriage status has been associated with cardiac disease (Das 2015; Gravel et al. 2015) and with higher risk of acute graft versus host disease in hematopoietic stem cell transplant recipients (Hill et al. 2017). Whether iciHHV-6 has additional consequences for human health is still unclear (Clark 2016; Collin and Flamand 2017). Likewise, it is presently unknown whether viral genetic determinants modulate disease presentation and geographic differences in clinical symptoms and epidemiology. Indeed, it was not until very recently that complete sequences for more than 180 HHV-6 genomes were obtained (Tweedy et al. 2016; Zhang et al. 2017; Greninger et al. 2018a,b; Telford, Navarro, and Santpere 2018). Analyses indicated that HHV-6A genomes are more diverse than HHV-6B (Telford et al. 2018) and that iciHHV-6A are highly divergent from exogenous HHV-6A viruses (Tweedy et al. 2016; Zhang et al. 2017). Several iciHHV-6B were found to be nearly identical, suggesting that they derived from the same integration event (Tweedy et al. 2016; Zhang et al. 2017; Greninger et al. 2018a). By mapping integration sites, Zhang et al indicated that this is the case for five iciHHV-6B sequenced from European subjects and estimated that their common ancestor existed long ago (∼24,000 years ago; Zhang et al. 2017).

Some level of geographic clustering was also reported for HHV-6A and -6B (Zhang et al. 2017; Greninger et al. 2018a; Telford et al. 2018), but the evolutionary history of these viruses has remained largely unexplored. Similarly, it is presently unknown whether interspecies recombination can occur in natural settings, as the only unequivocally defined interspecies recombinant is a laboratory strain (Greninger et al. 2018b).

## 2. Materials and Methods

### 2.1 Sequences, alignments, and similarity scores

We retrieved sequences of complete or almost complete HHV-6A and HHV-6B genomes from the NCBI database (http://www.ncbi.nlm.nih.gov/). Only one HHV-6 genome was retained from each set of inherited chromosomally integrated sequences derived from first-degree relatives (Greninger et al. 2018a), leading to a final set of 181 sequences (a list of NCBI accession number is reported in Supplementary Table S1).

HHV-6A strains included ten exogenous viruses and nineteen inherited chromosomally integrated sequences, whereas HHV-6B genomes were composed of sixty-eight viruses and eighty-four integrated genomes. Whole genome sequence alignments were generated using MAFFT (Katoh and Standley 2013) with the default parameters.

Pairwise identity scores were calculated as 1−(*M*/*N*) where *M* is the number of mismatching nucleotides and *N* the total number of positions along the alignment at which neither sequence has a gap character, as previously suggested (Muhire, Varsani, and Martin 2014). To make the analysis of all genomes computationally tractable, identity scores were calculated using the alignment of 181 HHV-6 genomes, rather than pairwise alignments (Supplementary Text S1).

Similarity plots of HHV-6 genomes were computed using a Kimura (two-parameter) distance model with SimPlot version 3.5.1 (Lole et al. 1999). The strip gap option was set at the 50% default value. Similarity scores were calculated in sliding windows of 1,000 bp moving with a step of 100 bp.

From complete genome alignments of HHV-6, HHV-6A, and HHV-6B sequences, 14,722, 4,687, and 6,102 parsimony-informative (PI) sites (sites that contain at least two types of nucleotides, each with a minimum frequency of two) were obtained, respectively. These sites were used as input for discriminant analysis of principal components (DAPC), linkage disequilibrium (LD), and population structure analyses.

### 2.2 Network construction and DAPC analysis

A neighbor-net split network of all whole genome sequences was constructed with SplitsTree v4.13.1 (Huson and Bryant 2006) using uncorrected p-distances and all polymorphic sites, after removing gap sites.

A DAPC (Jombart, Devillard, and Balloux 2010) was applied for all PIs the HHV-6 alignment. DAPC was selected because it allows the identification of clusters of genetically related individuals. Whereas approaches such as PCA (principal component analysis) describe the global diversity in a sample or population, in DAPC variance is partitioned into a between-cluster and within-cluster component. DAPC thus searches for synthetic variables (allele combinations) that maximize the variation among clusters while minimizing the variation within clusters. In DAPC, data are first transformed using PCA (to reduce the number of variables), the optimal number of clusters is identified, and then each sample is assigned to one of these clusters. The best number of clusters (*K* = 8) was identified through a Bayesian Information Criterion (Supplementary Fig. S1), using a sequential *K*-means clustering method with *K* from 1 to 15. After that, a discriminant analysis of the number of principal components that explained >95% of variance was applied, and clusters of the first and second linear discriminants were plotted. DAPC was carried out with the Adegenet R package (Jombart, 2008).

### 2.3 Recombination analysis

Recombination was evaluated using four methods implemented in RDP4 (RDP, GENECONV, MaxChi, and Chimera; Sawyer 1989; Smith 1992; Martin and Rybicki 2000; Posada and Crandall 2001; Martin et al. 2017). These methods were used because they showed good power in previous simulation analyses (Posada and Crandall 2001; Bay and Bielawski 2011).

In particular, the analysis was performed on the HHV-6 sequence alignment, after removing small repeats annotated as ‘rpt_type=TANDEM’ in either the HHV-6A or HHV-6B reference genomes (NC_001664 and NC_000898). To be conservative, only recombination events longer than 500 bp, with known parental sequences, and with a *P* value for all four methods < 0.01 were considered as significant. RDP4 was run with general default parameters and no permutations, by setting sequences as linear, by requiring topological evidence, and by checking alignment consistency. For the four methods, we applied default parameters were also used (RDP: widow size = 30; MaxChi: number of variable sites per window = 70, ‘strip gap’ option on; Chimera: number of variable sites per window = 60; GENECONV: ‘treat indel blocks as one polymorphism’ option on).

### 2.4 LD and population structure

LD—i.e. the non-random association of alleles at different polymorphic positions—was evaluated using the LIAN software v3.7 (Haubold and Hudson 2000). Briefly, LIAN tests for independent assortment by computing the number of loci at which each pair of haplotypes differs. From the distribution of mismatch values the program calculates a variance (*V*_D_), which is then compared with the variance expected under linkage equilibrium (*V*_e_). The null hypothesis that *V*_D_ = *V*_e_ can be tested by Monte Carlo simulation: the original dataset is scrambled by resampling the loci without replacement and for each resampled dataset, the *V*_D_ value is computed. The significance of the difference between *V*_D_ and *V*_e_ is calculated as the proportion of resampled datasets with a *V*_D_ value greater than or equal to that of the original dataset. We used this procedure with 1,000 iterations. LIAN also computes a standardized index of association (*I*_A_^S^), which is a measure of linkage and is based on the ratio between *V*_D_ and *V*_e_ scaled by the number of polymorphic positions. The *I*_A_^S^ is thus zero for linkage equilibrium.

We analyzed the population structure of HHV-6 using the program STRUCTURE (version 2.3) (Pritchard, Stephens, and Donnelly 2000). In general, population structure refers to a deviation from panmixia, whereby populations are somehow subdivided into subpopulations (e.g. due to geographic isolation). Very often subpopulations display differences in allele frequencies and the STRUCTURE method relies on a model in which the whole population is subdivided into *K* subpopulations characterized by a set of allele frequencies at each locus (Pritchard, Stephens, and Donnelly 2000). To run STRUCTURE, the allele frequency spectrum parameter (λ) was first estimated by using the ‘estimate λ’ model for *K* = 1, as suggested (Falush, Stephens, and Pritchard 2003): values of 0.60 (all HHV-6), 1.49 (HHV-6A), and 0.38 (HHV-6B) were obtained and used in the subsequent analyses. We next applied the linkage model with correlated allele frequencies, which extends the admixture model to (weakly) linked loci (Falush, Stephens, and Pritchard 2003). The admixture model with correlated frequencies allows for individuals to have mixed ancestry and assumes allele frequencies in closely related subpopulations to be similar because of migration or shared ancestry. Thus, this model has good power to detect subtle population structure (Falush, Stephens, and Pritchard 2003). The admixture model with correlated frequencies also assumes that all subpopulations diverged from a common ancestral population, which is characterized by a set of allele frequencies estimated by the model. The amount of drift that each subpopulation experienced from these ancestral frequencies is quantified by the *F* parameter, which is thus similar in concept to the fixation index (*F*_ST_), a measure of population differentiation based on allele frequencies.

To run STRUCTURE, map distances were set equal to PI site physical distances. The optimal number of populations was determined by running the model for *K* = 1–10. For each *K*, ten runs were performed with Markov chain Monte Carlo run lengths of 50,000 and 20,000 burn-in. Evanno’s method was used to select the optimal *K* (Evanno, Regnaut, and Goudet 2005). Results of independent runs were merged by permutating clusters using CLUMPAK (Kopelman et al. 2015) to generate the Q-value matrix.

To evaluate the contribution of the ancestral component to each PI site, a run with the optimal *K* was performed with the SITEBYSITE option selected.

### 2.5 Phylogenetic tree and nucleotide diversity

Phylogenetic trees were reconstructed using the phyML software using a general time reversible model plus gamma-distributed rates and four substitution rate categories (Guindon et al. 2009).

Nucleotide diversity on whole genome alignments was estimated using two parameters: the scaled number of segregating sites (θ_W_ (Watterson 1975)) and the average number of pairwise differences (π (Nei and Li 1979)). Tajima’s *D* (Tajima 1989) was also calculated. All analyses were performed using the POP-GENOME R package (Pfeifer et al. 2014).

## 3. Results

### 3.1 Phylogenetic relationships and DAPC

We obtained a list of complete or almost complete HHV-6 genomes from public databases. These 181 genomes (29 classified as HHV-6A and 152 as HHV-6B) were aligned and a neighbor-net split network was generated. As expected, HHV-6A and -6B sequences were clearly separated in the network (Fig. 1A). HHV-6A sequences showed higher genetic diversity, especially between iciHHV-6A and exogenous viruses, whereas most HHV-6B genomes were very closely related and clustered together. However, some HHV-6B exogenous viral sequences diverged from all other HHV-6B genomes. All these divergent viruses were sampled in the 90s, in New York state (Rochester), from children with acute febrile illness and different ethnic background (Greninger et al. 2018a).

**Figure 1.** HHV-6 divergence. (A) Neighbor-net split network of 181 HHV-6 genome sequences. Each sample is shown as a dot and colors are indicated in the legend. Divergent HHV-6B exogenous viral sequences sampled in New York state are labeled. (B) DAPC of HHV-6 genomes. The first two discriminants are plotted and samples are colored as in panel A. For each cluster, values of nucleotide diversity (θ_W_, π) and Tajima’s D are also reported. vHHV-6A: HHV-6A exogenous virus; iciHHV-6: inherited chromosomally integrated HHV-6; NY cluster: New York HHV-6B cluster.

To gain further insight into the structure of HHV6 populations, we applied a DAPC. This approach can identify the principal components that explain most between‐group variation while minimizing within‐group variation (Jombart, Devillard, and Balloux 2010).

Results showed the presence of four major clusters, reflecting the neighbor-net split network (Fig. 1B). HHV-6A and HHV-6B were clearly separated, with the former generating two distinct clusters, one composed of iciHHV-6A sequences, and the other including exogenous viruses only. The HHV-6A virus cluster showed less variability compared with the iciHHV-6A one. Conversely, most of HHV-6B genomes, both integrated copies and exogenous viruses, clustered together, with the exception of fifteen viral samples (Fig. 1B). All these genomes correspond to those that showed high divergence in the network analysis (Fig. 1A), and form a separate cluster, which is hereafter referred to as the NY cluster after the place of their sampling (Fig. 1B).

We next calculated pairwise identity scores for the 181 genomes. In particular, identity scores were computed as the percentage of matching nucleotides over the total number of positions along the alignment at which neither sequence has a gap character, as suggested (Muhire, Varsani, and Martin 2014). This approach also avoids deflation of identity scores for sequences with missing information (partial genomes). Pairwise identity scores clearly separated HHV-6A and HHV-6B sequences (Fig. 2A). NY cluster sequences, however, showed variable levels of identity to other HHV-6B genomes and, compared with the latter, higher similarity to HHV-6A sequences. In line with the DAPC results, NY cluster and HHV-6B sequences were relatively homogeneous, whereas HHV-6A genomes showed higher diversity (Fig. 2A).

**Figure 2.** HHV-6 sequence identity. (A) Color-coded pairwise identity matrix generated from 181 HHV-6 genomes. Each cell represents the percentage identity score between two sequences (indicated horizontally and vertically). The legend indicates the correspondence between pairwise identities and the color code. Identity scores were computed over all positions where gaps are not observed in either sequence (see Section 2). iciHHV-6: inherited chromosomally integrated HHV-6; vHHV-6: exogenous HHV-6 viruses; the number of genomes (n) is also reported. (B) Similarity plot (generated with SimPlot) of representative NY cluster, HHV-6A, and HHV-6B genomes to the HHV-6A reference genome (U1102 strain). Each curve represents the comparison between a genome and the reference. Similarity (Kimura distance) was calculated within sliding windows of 1,000 bp moving with a step of 100 bp. The missing information for NY cluster viruses in the 5′ and 3′ genome regions is due to poor coverage (partial genome sequencing). A schematic representation of the HHV-6 genome is also shown. The positions (relative to the genome alignment) of the left and right DRs, of the origin of replication (*ori*Lyt), as well as of the intermediate repeats (R1, R2, and R3) are reported.

A sliding window analysis of sequence similarity was performed by comparing five NY cluster viruses, as well as HHV-6B and HHV-6A genomes, to the HHV-6A reference sequence (U1102 strain). These genomes were selected as representatives of the respective groups. Plots revealed multiple genomic regions where, compared with other HHV-6B sequences, NY cluster viruses showed higher similarity to the U1102 strain (Fig. 2B). This was particularly evident in two relatively large and continuous genome segments (Fig. 2B).

HHV-6B genomes have nine open reading frames (ORFs) (originally referred to as B1–B9) that are not shared with HHV-6A (Dominguez et al. 1999). The genomic regions where ORFs B1-B5 and B9 are located are poorly covered in samples from New York state (as several of these genomes lack sequence information at the 5′ and 3′ genome ends). We however inspected B6, B7 and B8 sequences in NY cluster genomes. Alignment of B6 sequences indicated that all NY cluster genomes possess the initial methionine (which is absent exogenous HHV-6A viruses), but at least for those showing no sequencing uncertainties, two single nucleotide insertions, also observed in HHV-6A genomes, prevent translation of the complete protein (Supplementary Text S2). A similar situation is observed for B7, whereby NY cluster and HHV-6A sequences carry a di-nucleotide insertion that disrupts the reading frame (Supplementary Text S2). Finally, in the case of B8, NY cluster viruses are variable with respect to the presence of an ATG initiation codon (which is present in HHV-6B), but all carry a single nucleotide deletion that causes the creation of a premature STOP codon (Supplementary Text S2). Thus, at least for NY cluster viruses with no sequence uncertainties, the predicted coding potential does not include the B6–B8 ORFs, which are instead complete in other viruses sampled in New York state but not belonging to the NY cluster.

The possibility that NY cluster genomes represent sequencing artifacts (mixed assemblies) deriving from individuals infected with HHV-6A and HHV-6B was considered very unlikely based on the percentage of reads mapping to HHV-6A and HHV-6B genomes, which was definitely skewed towards HHV-6B and in any case comparable to other genomes sequenced from New York state samples but clustering with HHV-6B genomes (Supplementary Table S2). We thus reasoned that NY cluster sequences may derive from interspecies recombination events.

### 3.2 LD and recombination

Intraspecies recombination was previously documented for HHV-6 (Greninger et al. 2018a; Telford et al. 2018), whereas only one interspecies recombinant (the DA strain) has been reported to date and proposed to have originated via co-culturing of HHV-6A and -6B viruses (Greninger et al. 2018b). We thus first analyzed the level of LD with LIAN v3.7, which tests the null hypothesis of linkage equilibrium across loci (Haubold and Hudson 2000). Statistically significant LD was detected for both HHV-6A and HHV-6B sequences (Monte Carlo simulations, 1,000 repetitions, *P* < 10^−^^3^). However, the standardized index of association (*I*_A_^S^) resulted equal to 0.199 for HHV-6A and 0.204 for HHV-6B. These values indicate low to moderate LD and, therefore, they are consistent with some level of recombination. As expected, LD was higher when HHV-6A and -6B were analyzed together (*I*_A_^S =^ 0.395).

We next directly explored whether interspecies recombination occurred and if this phenomenon originated the NY cluster. We used four methods implemented in the RDP4 software. To be conservative, we only retained recombination events longer than 500 bp and with known parental sequences. A total of nineteen unique recombination events were detected and twelve of them were interspecies (Table 1 and Supplementary Table S3). Among these latter, we detected the previously described recombination event involving the DA strain. All other interspecies recombinants belonged to NY cluster viruses, which were apparently involved in multiple distinct recombination events with HHV-6A sequences (Table 1). However, RDP4 was unable to determine whether the parentals were iciHHV-6A or exogenous HHV-6A viruses. Moreover, not all NY cluster sequences were identified as recombinants.

**Table 1.** Interspecies recombination events.

	Start*	End*	Recombinant sequence	Minor parental sequence (*n*^a^)	Major parental sequence (*n*^a^)	
1	20,053	20,834	NY-390	vHHV-6A (7)	vHHV-6B (53)	
				iciHHV-6A (19)	iciHHV-6B (84)	
2	67,524	72,695	DA	vHHV-6B (60)	vHHV-6A (7)	
				NY cluster (15)	iciHHV-6A (19)	
				iciHHV-6B (74)		
3	68,313	68,983	NY-390	vHHV-6A (1)	vHHV-6B (50)	
				iciHHV-6A (5)	iciHHV-6B (84)	
4	68,313	69,067	NY-338	vHHV-6A (1)	vHHV-6B (49)	
				iciHHV-6A (6)	iciHHV-6B (84)	
5	68,327	68,729	NY-129; NY-350	vHHV-6A (1)	vHHV-6B (52)	
				iciHHV-6A (5)	iciHHV-6B (85)	
6	68,326	69,067	NY-379	vHHV-6A (1)	vHHV-6B (49)	
				iciHHV-6A (5)	iciHHV-6B (84)	
7	75,608	76,583	NY-390; NY-350	vHHV-6A (10)	vHHV-6B (53)	
				iciHHV-6A (19)	NY-cluster (9)	
					iciHHV-6B (85)	
8	75,608	76,841	NY-379	vHHV-6A (10)	vHHV-6B (53)	
				iciHHV-6A (11)	NY-cluster (7)	
					iciHHV-6B (85)	
9	119,809	120,946	NY-241; NY-350	vHHV-6A (3)	NY-cluster (3)	
				iciHHV-6A (1)		
10	125,850	137,218	NY-379	vHHV-6A (3)	NY-cluster (1)	
				iciHHV-6A (3)		
11	137,530	141,294	NY-338, NY-379	vHHV-6A (6)	vHHV-6B (1)	
				iciHHV-6A (12)		
12	149,095	150,089	NY-241; NY-338; NY-350	vHHV-6A (10)	NY-cluster (1)	

Note: *Positions refer to U1102 sequence (NC_001664). Recombination events are mapped onto genomic structures in Fig. 4. iciHHV-6: inherited chromosomally integrated HHV-6; vHHV-6: exogenous HHV-6 viruses; NY-cluster: New York HHV-6B cluster.

a Number of sequences identified as possible parentals by RDP4.

### 3.3 Population structure analysis

To gain further insight into the evolutionary origin of HHV-6A and HHV-6B genomes, we investigated the ancestry and admixture of HHV-6 using the STRUCTURE program, which relies on a Bayesian statistical model for clustering genotypes into populations without prior information on their genetic relatedness or geographic origin. STRUCTURE can identify distinct subpopulations (or clusters, *K*) that compose the overall population and assigns each individual to one or more of those clusters. Initially, the 181 HHV-6A and -6B genomes were used for STRUCTURE analysis with correlated allele frequencies under the linkage model (Pritchard et al. 2000; Falush, Stephens, and Pritchard 2003). This model, which is well-suited for markers that are weakly linked (Falush, Stephens, and Pritchard 2003), uses LD among loci and assumes that discrete genome ‘chunks’ are inherited from ancestral populations.

The optimal number of subpopulations (*K*) was estimated to be equal to 2 and STRUCTURE clearly separated the HHV-6A and HHV-6B ancestry components (Fig. 3A and Supplementary Fig. S2). In line with the recombination analysis, sequences from the NY cluster had a proportion of their ancestry from the HHV-6A subpopulation. However, the HHV-6A ancestry component was evident in all NY cluster sequences and not only in those identified as recombinants (Fig. 3A, Table 1).

**Figure 3.** HHV-6 population structure. (A) Bar plot representing the proportion of ancestral population components from the STRUCTURE linkage model for HHV-6, HHV-6A, and HHV-6B. Each vertical line represents a HHV-6 genome. Samples are ordered on the basis of their integration/exogenous status, of viral species classification, and of geographic origin. Stars indicate European iciHHV-6B sequences deriving from the same integration event (Zhang et al. 2017). (B) Distributions of posterior *F* values for the ancestral populations. Colors are as in panel (A).

The linkage model also provides information on the level of drift of each subpopulation from a hypothetical common ancestral population. In particular, STRUCTURE estimates the *F* parameter, which represents a measure of genetic differentiation between populations based on allele frequencies (see Section 2). The *F* value for the HHV-6A component was substantially lower than that of the HHV-6B component (Fig. 3B), indicating that HHV-6A genomes diverged less than HHV-6B genomes from the ancestral common HHV-6A/B population.

The strong genetic differentiation between the HHV-6A and -6B populations may mask further sub-level clustering. Thus, STRUCTURE analysis was repeated for HHV-6A and HHV-6B genomes separately.

For HHV-6A, the best *K* resulted equal to 4 (Supplementary Fig. S2). Analysis of ancestry components indicated that a large proportion (almost 100% for non-African viruses) of exogenous viral genomes was contributed by a single ancestral population (population HHV-6A-1, Fig. 3A) that is virtually absent in iciHHV-6A. These latter showed limited evidence of geographic structure and variable levels of admixture among three ancestral populations, with the exclusion of the two Asian sequences, which had a major proportion of their ancestry from a single population (population HHV-6A-2, Fig. 3A). In turn, population HHV-6A-2 contributed a proportion of ancestry to iciHHV-6A sampled in Europe and America, as well as to African HHV-6A viruses. The *F* value for population HHV-6A-2 was substantially lower than those for the three other populations (Fig. 3B). The homogeneous ancestry of European and American exogenous viruses suggests the population underwent a bottleneck. Overall, these results are consistent with the DAPC and splits-tree analysis by showing that HHV-6A exogenous viruses and iciHHV-6A are divergent and derived most of their genomes from distinct ancestral populations.

In the case of HHV-6B, the best number of cluster was estimated to be 3 (Supplementary Fig. S2). The three ancestral components (populations HHV6B-1 to -3) were represented both in exogenous viruses and in iciHHV-6B, although with different proportions (Fig. 3A). Viruses belonging to the NY cluster displayed a high proportion of ancestry from population HHV-6B-1, which is thus expected to comprise the HHV-6A component and had, in fact, the lowest *F* value (Fig. 3B). Apart from the NY cluster, exogenous viral and iciHHV-6B populations were similar in terms of ancestry components, and no overt geographic structure was observed. Most iciHHV-6B sampled in Europe and USA showed similar and low levels of admixture. These included the five European iciHHV-6B sequences deriving from the same integration event (Zhang et al. 2017). The major ancestry component of these genomes, as well as of most other iciHHV-6B, was the one with the highest *F* value (HHV-6B-3; Fig. 3B). This suggests that the exogenous viral populations that integrated into these chromosomes had already drifted away from the ancestral population, most likely as the result of one of more bottlenecks. The component with intermediate *F* values (HHV-6B-2) was most abundant in exogenous viruses samples in Asia and Africa, as well as in iciHHV-6B from Asian individuals.

### 3.4 Analysis of ancestry components and recombination events

To gain further insight into the interspecies recombination events and ancestry components, we exploited the site-by-site inference in STRUCTURE, which allows population-of-origin assignment for individual variants. This is achieved by the linkage model, which exploits LD among loci to infer which genome chunks were derived from which ancestral population (Falush, Stephens, and Pritchard 2003).

As expected, for NY cluster viruses, the HHV-6A ancestry component from the HHV-6A plus HHV-6B analysis overlapped with the most ancestral component from the HHV-6B only analysis (population HHV-6B-1) (Fig. 4). This is in line with the *F* value analysis reported earlier and indicates that the HHV-6B-1 component, which accounts for a large proportion of NY cluster genomes (Fig. 3A), indeed comprises the HHV-6A component. Recombination events also overlapped remarkably well with these components. However, the ancestry proportions of NY cluster viruses could not be fully explained by recombination events (Fig. 4).

**Figure 4.** Ancestral components of NY cluster viruses. Site by site probability for the HHV-6A (A) and the HHV-6B-1 (B) ancestry components. Each line represent a NY cluster virus genome and each dot represents a SNP with a *P* > 0.80 to derive from the HHV-6A ancestry component (red) or the HHV-6B-1 ancestry component (green). Colors are the same as in Fig. 3. All the recombination events involving NY cluster viruses are also reported (see Table 1). Positions refer to HHV-6 and HHV-6B alignments, respectively. A schematic representation of HHV-6 genomes is also shown with landmark elements as in Fig. 2B.

Because, according to RDP4, not all NY cluster viruses were involved in recombination events, but all share similar proportions of HHV-6A ancestry, we used a maximum likelihood approach to reconstruct the phylogenies of the two largest regions involved in recombination events (events ten and eleven in Fig. 4). Results indicated that, for both regions, the NY cluster viruses detected as recombinants were more closely related to HHV-6A than to HHV-6B sequences (Fig. 5). However, the remaining members of the NY cluster showed variable levels of divergence from each other and from HHV-6A and -6B sequences. For these genomic regions, the divergence of iciHHV-6A and exogenous -6A viruses was also blurred, explaining why RDP4 was unable to infer the parental genome as either iciHHV-6A or exogenous HHV-6A. Importantly, the branching patterns of the NY cluster sequences were inconsistent with the hypothesis that they derived from recent recombination of known HHV-6B and -6A genomes. By taking into account STRUCTURE results, at least two scenarios can be envisaged to explain these findings: 1) that the NY cluster population progressively diverged from an ancestral HHV-6A-like population and a recent bottleneck originated the large HHV-6B cluster; 2) that ancient recombination events between ancestral HHV-6A and -6B populations originated the NY cluster population, which subsequently underwent a bottleneck resulting in most HHV-6B sequences sampled to date. The second scenario, however does not explain why virtually no HHV-6B-derived component is observed in HHV-6A populations.

**Figure 5.** Phylogenetic trees of putative recombinant regions in NY cluster strains. (A) Maximum likelihood tree generated using the multiple sequence alignment (length = 15,213 bp) of the genomic region found to be involved in recombination event ten (Table 1). (B) The same as in (A) for the genomic region involved in recombination event eleven (alignment length = 5,706 bp). The specific sequences that were identified as recombinants (Table 1) are indicated on the tree. Each dot represents a sample and colors are shown in the legend.

### 3.5 Levels and patterns of intraspecies polymorphism

Finally, to further investigate the evolutionary history of HHV-6A and -6B, the level of intraspecies polymorphism was examined by estimating genetic diversity (Θ_w_ and π) at all polymorphic sites (Watterson 1975; Nei and Li 1979). Tajima’s *D* (Tajima 1989) was also calculated. *D* values close to zero are expected in neutrally evolving populations of constant size, whereas positive values derive from an excess of intermediate frequency variants, due to balancing selection or population shrinkage. Negative Tajima’s *D* values indicate an excess of low frequency polymorphism caused either by background selection, selective sweep or population expansion. Although the effect of demography and selection are difficult to disentangle, selective events usually affect a relatively small fraction of sites and genome-wide estimates are thus more likely to be indicative of demographic forces acting on the population.

The highest nucleotide diversity was observed for the NY cluster and for iciHHV-6A (Fig. 1B). These populations had positive values of Tajima’s *D* relatively close to 0, suggesting almost constant population size. HHV-6A exogenous viruses also had relatively high levels of polymorphism; taking the STRUCTURE results into account, this is likely contributed by the African viruses. Nonetheless, Tajima’s *D* was negative, suggesting that the European and American viruses underwent a bottleneck and recent population expansion. Finally, iciHHV-6B and exogenous HHV-6B viruses not belonging to the NY cluster had low diversity and negative *D* values (Fig. 1B). Again is accordance with STRUCTURE inference, these populations most likely underwent one or more bottleneck followed by population expansion.

## 4. Discussion

Roseolovirus infection is ubiquitous and poses an important burden on human health (Hill and Zerr 2014; Tesini, Epstein, and Caserta 2014). Investigation of viral genetic determinants as possible modulators of disease presentation has not been undertaken and most clinical and epidemiological studies only categorize infection as being HHV-6A or -6B. This is partially because the genomics of roseoloviruses has lagged behind compared with that of other herpesviuses and a sizable number of HHV-6 genomes, either from clinical samples or integrated in human chromosomes, was made available only recently (Tweedy et al. 2016; Zhang et al. 2017; Greninger et al. 2018a,b; Telford et al. 2018). Herein, we used these sequence data to investigate the evolutionary relationships between HHV-6A and -6B, to analyze their genetic diversity and geographic structure (or lack thereof), as well as to assess whether interspecies recombination occurs in natural settings.

In line with previous data, most analyses clearly differentiated HHV-6A and -6B sequences (Tweedy et al. 2016; Zhang et al. 2017; Greninger et al. 2018a,b; Telford et al. 2018). Nonetheless, the neighbor-net split network and DAPC analyses detected the NY cluster as a viral population distinct from the majority of HHV-6B sequences. The initial hypothesis that these genomes derived from recent interspecies recombination was supported by RDP4 analysis, which identified multiple recombination events between HHV-6A and -6B sequences that involved NY cluster viruses. However, STRUCTURE analysis and closer inspection of the results indicated that not all NY viruses were identified as recombinants and that the HHV-6A ancestry component was not only detected in regions involved in recombination events. Although the lack of recombination signals for some sequences and regions may be due to the fact that the events were ancient and followed by divergence, phylogenetic analysis of the recombinant fragments indicated that NY cluster sequences formed multiple internal branches and showed variable levels of divergence among themselves and from HHV-6A and -6B. This pattern is not consistent with ancient recombination events, as divergence from a common branch would be expected if this were the case.

STRUCTURE analysis estimated that HHV-6A genomes diverged less from a common ancestral population than -6B genomes. Consistently, the HHV-6B-1 ancestry component, which is most abundant in NY cluster sequences and which comprises the HHV-6A component, had lower *F* values compared with the other HHV-6B components. Thus, HHV-6B genomes other than the NY cluster experienced stronger drift, possibly because of a bottleneck with subsequent population expansion that resulted in loss of diversity. This view is also supported by calculation of nucleotide diversity and Tajima’s *D*. Thus, the detected recombination events represent shared ancestry between NY cluster viruses and HHV-6A populations, and the recent divergence of most HHV-6B genomes from HHV-6A sequences possibly originated the spurious signals.

Overall, we consider that the most likely scenario envisages the presence of an ancestral HHV-6A-like population from which HHV-6A sequences and the NY cluster population diverged. A relatively recent bottleneck of the NY (or a related) population with subsequent expansion originated most HHV-6B genomes sampled to date. Based on the plausible assumption that iciHHV-6 have the same mutation rate as the human genome, Zhang et al. (2017) estimated that the integration event of a subset of identical iciHHV6B in Europeans occurred around 24,000 years ago. It follows that the events that led to the divergence of HHV-6A and -6B viruses, as well as of the NY cluster, occurred in a distant past.

Estimates of iciHHV-6 carriage status indicated that the frequency of iciHHV-6B is higher than that of iciHHV-6A (Clark 2016). Recent work showed that HHV-6A and -6B laboratory strains have similar chromosomal integration efficiency. Nonetheless, differences were observed depending on the cell-type, raising the possibility that the ability to infect germs cells may be different for HHV-6A and -6B (Gravel et al. 2017). At present, it is unknown which fraction of iciHHV-6 derive from founder effects. Beside the above-mentioned European iciHHV-6B sequences, other authors have indicated that multiple HHV-6 sequences derived from ancestral integrations (Kawamura et al. 2017). Data herein do not address this question, nor elucidate the frequency with which HHV-6 can integrate and be transmitted vertically. STRUCTURE data however indicate that currently sequenced iciHHV-6A derive from viral populations that experienced limited drift compared with iciHHV-6B and are, therefore, most likely older. Indeed, iciHHV-6A are diverse and possibly represent a snapshot of integration events that involved extinct or still unsampled viral populations. Extant exogenous HHV-6A viruses, especially those sampled outside Africa, have a large fraction of their ancestry deriving from a population that is not represented in iciHHV-6A. This does not necessarily imply that modern HHV-6A viral populations have reduced integration efficiency, but might instead reflect a sampling bias. Notably, this situation is the opposite than that of HHV-6B, whereby integrated copies reflect viral populations responsible for active infections in the same areas. The exception is represented by NY cluster viruses, as no iciHHV-6B is closely related to this population. Again, this might be due to the biased geographic origin of most iciHHV-6B sequences. The sampling of all NY cluster viruses in the USA does not necessarily mean that they have long-standing association with the American continent, as both past and recent human migrations may have introduced the viruses from other locations. Thus, NY cluster viruses might have integrated in the (presently unsampled) genomes of populations living where these viruses are endemic. Therefore, our data do not explain geographic differences in iciHHV-6 carriage status, which is reportedly lower in Africa and Asia than it is in Europe and North America (Clark 2016; Tweedy et al. 2016). However, both for iciHHV-6A and -6B, European and American sequences tend to have high proportions of ancestry from viral populations that experienced considerable drift. A possible interpretation is that environmental, behavioral, demographic, or genetic factors increased infection rates among early Europeans and consequently determined faster changes in viral genetic composition and higher chances for integration. The testing of this and other hypotheses on the geographic origin and spread of HHV-6 will necessarily require the sequencing of additional integrated and exogenous genomes. Indeed, the recent sampling of NY cluster viruses suggests that diverse HHV-6 populations exist.

For these very reasons, our study has limitations that include the relatively low number of available HHV-6A sequences and the skewed sampling of both HHV-6A and -6B in terms of geographic locations. Several geographic areas and human ethnic groups or communities are not represented at all or are represented by very few sequences (e.g. Central and Southern Asia, Native Americans, and Native Austronesians). As for Sub-Saharan Africa, where HHV-6 was previously suggested to have originated (Tweedy et al. 2016), few exogenous viruses and only one iciHHV-6A were sequenced. The sampling in Asia is also relatively sparse. Nonetheless, twenty HHV-6B exogenous viruses were available for Japan, where the virus represents the second most common cause of infection-related encephalitis (Hoshino et al. 2012). The proportions of ancestry components of these viruses tended to differ from most of those sampled in the USA, although it is presently impossible to determine whether these differences account for distinct clinical symptoms. Likewise, the clinical consequence of NY cluster virus infection is presently unknown, as no detailed information was provided for the patients from whom these sequences were obtained. These viruses have a consistent HHV-6A-like ancestry component and, in a marmoset model, HHV-6A was found to display higher neuropathogenicity than HHV-6B (Leibovitch et al. 2013). *In vitro* studies showed that HHV-6A, but not HHV-6B, productively infects glial cells (Donati et al. 2005; Harberts et al. 2011; Reynaud et al. 2014). In mouse models, HHV-6A DNA persists for months in the brain, whereas HHV-6B DNA levels decreased rapidly after infection (Reynaud et al. 2014). HHV-6A and -6B also differ in terms of sensitivity to Type I interferons, distribution in human tissues, immunological properties, and in other biomedical aspects (Jaworska, Gravel, and Flamand 2010; Ablashi et al. 2014). These distinctions were indeed considered as supportive of the classification of HHV-6 into the two species (Ablashi et al. 2014). Data herein indicate that the evolutionary relationships between HHV-6A and -6B are more complex than previously thought. NY cluster viruses display higher similarity to HHV-6A than most HHV-6B sequences. It is therefore difficult to establish, based on sequence data alone, whether these viruses should be classified as HHV-6A or HHV-6B. Assuming that the reported differences between HHV-6A and -6B are caused by viral genetic determinants, our data indicate that the phenotype of NY cluster viruses might be distinct from either HHV-6B or HHV-6A or both, irrespective of how they are formally classified. More generally, future efforts to determine and map the genetic determinants of HHV-6 phenotypes will be of central importance to understand the pathogenic potential of these ubiquitous infectious agents.

## Data availability

A list of NCBI accession number of all sequences analyzed is reported in Supplementary Table S1.

The alignment of 181 HHV-6 genomes is available as Supplementary Text S1.

## Funding

This work was supported by the Italian Ministry of Health, grant number RC 2019 to M.S. and RC 2018–2019 to D.F.

**Conflict of interest:** None declared.

## Supplementary Material

vez043_Supplementary_Data
